# Adoption of Snake Variable Model-Based Method in Segmentation and Quantitative Calculation of Cardiac Ultrasound Medical Images

This article has been retracted.

**DOI:** 10.1155/2021/2425482

**Published:** 2021-07-26

**Authors:** Xing Huang, Haozhi Zhu, Jiexin Wang

**Affiliations:** Department of Ultrasound, Affiliated Hospital of Guangdong Medical University, Zhanjiang 524001, Guangdong, China

## Abstract

This paper intends to explore the effect of the enhanced snake variable model in the segmentation of cardiac ultrasound images and its adoption in quantitative measurement of cardiac cavity. First, the basic principles of the traditional snake model and the gradient vector flow (GVF) snake model are explained. Then, an ellipsoid model is constructed to obtain the initial contour of the heart based on the three-dimensional volume of cardiac ultrasound image, and a discretized triangular mesh model is generated. Finally, the vortical gradient vector flow (VGVF) external force field is introduced and combined with the greedy algorithm to process the deformation of the initial ellipsoid contour of the heart. The segmentation effect is quantitatively evaluated regarding the area overlap rate (AOR) and the mean contour distance (MCD). The results show that the VGVF snake model can segment the deep recessed area of the “U-shaped map” in contrast to the traditional snake model and the GVF snake model. After being applied to ultrasonic image segmentation, the VGVF snake model obtains the segmentation result that is close to the doctor's manual segmentation result, and the average AOR and MCD are 97.4% and 3.2, respectively. The quantitative evaluation of the cardiac cavity is carried out based on the segmentation results, and the measurement of the volume change of the left ventricle within a cardiac cycle is realized. To sum up, VGVF snake model is superior to the traditional snake and GVF snake models in terms of ultrasonic image segmentation, which realizes the three-dimensional segmentation and quantitative calculation of the cardiac cavity.

## 1. Introduction

In the field of modern medicine, imaging information has become an indispensable tool for diagnosis, treatment, and research. Medical imaging information can intuitively reflect the characteristics of human organs/tissues, such as morphology, function, and pathological changes [1, 2]. Ultrasonic medical imaging-assisted diagnosis technology has the advantages of noninvasive, nondamaging, and nonionizing radiation and has become an important tool in clinical diagnosis and treatment [3]. In cardiovascular ultrasound diagnosis and treatment, the morphological characteristics of the heart are important information for detection, such as the heart wall thickness, transverse diameter, motion range, and anatomical structure. Through such information, the diagnosis of cardiovascular diseases can be achieved efficiently [4]. Motion tracking, three-dimensional reconstruction, and functional mapping registration in computer-aided diagnosis technology are all important components of current cardiovascular ultrasound medical diagnosis [5]. Image segmentation is an indispensable step for providing raw data in the image analysis process, which includes feature selection and extraction. The purpose of image segmentation is accurately extracting useful feature information in a noisy environment [6].

The snake model utilizes the high-level information in the image to minimize energy to solve machine vision problems. Snake model has been widely used in auxiliary extraction of image features, target segmentation, tracking of moving targets, etc., and provides reliable segmentation results for target edge detection, video matching, and image 3D reconstruction. For example, Chen et al. [7] used the snake model and the GVF snake model to segment ultrasound images. The GVF snake model had better noise resistance and convergence characteristics compared with the snake model. Yan et al. [8] used the snake model to segment the ultrasound image surgical instruments during surgery [8]. However, this model has problems such as initialization and poor segmentation of recessed areas [9–11]. Since the structure of human organs and tissues is relatively complex, problems such as sound wave signal interference can affect the quality of ultrasound imaging, and artifacts or noise are ultimately generated in the image, which seriously affects the robustness of segmentation [12].

Based on the above issues, the basic principles of the traditional snake model and the gradient vector flow (GVF) snake model are explained. VGVF external force field and greedy algorithm are introduced in the segmentation of cardiac ultrasound images to improve the segmentation effect. Quantitative indexes are used to compare the differences in the segmentation of cardiac cavity by different models. Moreover, a quantitative calculation of the volume change of the left ventricular cavity is performed based on the results of the segmentation of the cardiac cavity. This study intends to provide a reference for improving the segmentation effect of cardiac ultrasound images.

## 2. Basic Principles

### 2.1. The Basic Principles of the Traditional Snake Model

Snake model is also called active contour model. The mathematical expression of parametrics is *X*(*s*) = [*x*(*s*), *y*(*s*)], *s *∈* *[0, 1], where *x*(*s*) and *y*(*s*) represent the coordinate positions in the image where different control points are located, which are also the Fourier description form of the target contour. Snake model can act and move in the image space to form a closed curve by using the internal energy of the curve itself and the image energy [13]. Snake model searches for the boundary or region of interest (ROI) in the image, which is the process of finding the energy minimum curve. There are many ways of image energy in the traditional snake model, and the problem of minimizing image energy can be transformed into a problem of solving functional extremum [14].

The advantages of the snake model are as follows: (i) the model is active, which can minimize energy and display its dynamic characteristics in real time; (ii) the model is interactive, and it can be manually intervened to find the boundary in any area; and (iii) the model is high-level information-oriented, which can take high-level energy information as a guide to search and locate energy minimization.

The snake model is defined as a curve *x*(*s*) = [*x*(*s*), *y*(*s*)] on the image plane *I*(*x*, *y*), where *I*(*x*, *y*) is the gray level in the original image, and *s* is the normalized form of the arc length parameter of the current position and *s* ∈ [0, 1]. Usually, the energy in the snake model is obtained by the addition of multiple values, which is conducive to the addition of energy constraints, and the energy mathematical expression of the snake model is as follows:

(1) $$\begin{array}{c} E\left(x\left(s\right)\right)=\int_{0}^{1}E_{\mathrm{int}}\left(x\left(s\right)\right)+E_{\mathrm{ext}}\left(x\left(s\right)\right)ds. \end{array}$$

The mathematical expression of the internal energy term determined by the nature of the curve is as follows:

(2) $$\begin{array}{c} E_{\mathrm{int}}=\frac{\alpha {\left|x^{\prime }\left(s\right)\right|}^{2}+\beta {\left|x^{\prime \prime }\left(s\right)\right|}^{2}}{2}. \end{array}$$

In equation (1) and equation (2), *E*_ext_ is the external image energy term and *E*_int_ is the internal image energy term. *x*′(*s*) and *x*^″^(*s*) are the first-order and second-order partial derivative of *x*(*s*), respectively. *α*|*x*′(*s*)|^2^ is the elastic internal energy (i.e., the elastic energy of the continuous and stretched edge points of the contour during the deformation process), and *α* is the elastic parameter. *β*|*x*^″^(*s*)|^2^ is the rigid internal energy (i.e., the smoothness and bendability characteristics of the contour curve in the evolution and convergence process), and *β* is a rigid parameter.

The external image energy term *E*_ext_ is produced by external forces, which is produced in many forms, such as line energy *E*_line_, edge energy *E*_edge_, and termination energy *E*_trem_. The mathematical expressions for different energies are as follows:

(3) $$\begin{array}{c} \left\{\begin{array}{c} E_{\text{line}}=-{\left(G_{\sigma }*\nabla^{2}I\right)}^{2},\\ E_{\text{edge}}=-{\left|\nabla I\left(x,y\right)\right|}^{2},\\ E_{\text{term}}=\frac{\partial^{2}C/\partial n_{⊥}^{2}}{\partial C/\partial n}. \end{array}\right. \end{array}$$

In equation (3), *σ* is the standard deviation, *G*_*σ*_ is the two-dimensional Gaussian function, ^*∗*^ is the convolution operator of the two-dimensional image, and ∇ is the gradient operator.

Snake model is leaded to deform, so as to realize task segmentation, which is also the process of minimizing energy. When *E*(*x*(*s*)) is located on a certain curve and obtains an extreme value, the following equation can satisfy Euler's equation:

(4) $$\begin{array}{c} \alpha x^{\prime }\left(s\right)+\beta x^{\prime \prime \prime }\left(s\right)-\nabla E_{\text{ext}}=0. \end{array}$$

Therefore, the problem of energy minimization is transformed into the problem of solving partial differential equations, which belongs to the boundary value problem, and a variety of boundary value conditions can be set. To satisfy the snake profile as a closed curve, the boundary value condition is usually set as *x*(0) = *x*(*n*). If the snake model is regarded as a function of time, it can be solved using the finite difference iteration method and force balance equation as follows:

(5) $$\begin{array}{c} x\left(s,t\right)=\alpha x^{\prime \prime }\left(s,t\right)+\beta x^{\prime \prime \prime }\left(s,t\right)-\nabla E_{\text{ext}},\\ F_{\mathrm{int}}+F_{\text{ext}}=0. \end{array}$$

### 2.2. The Basic Principles of the GVF Snake Model

The Gaussian convolution in the traditional snake model can appropriately expand the initialization range, but it can only be effective at or near the boundary of the image, so this model has the problem of not being able to enter the “recessed” area. GVF snake model is a novel external force field model. The external force field of the model is only obtained by adding it to the force balance equation after calculation, which makes the model have dynamic significance [15]. The mathematical expression of the GVF snake model is as follows:

(6) $$\begin{array}{c} x\left(s,t\right)=\alpha x^{\prime \prime }\left(s,t\right)+\beta x^{\prime \prime \prime }\left(s,t\right)-U. \end{array}$$

In equation (6), *U*(*x*, *y*)=[*u*(*x*, *y*), *v*(*x*, *y*)] is a vector, which is obtained by calculating the functional extremum of the integral equation.

(7) $$\begin{array}{c} \varepsilon =\iint \mu \left(u_{x}^{2}+u_{y}^{2}+v_{x}^{2}+v_{y}^{2}\right)+{\left|\nabla f\right|}^{2}{\left|U-\nabla f\right|}^{2}dxdy. \end{array}$$

In equation (7), *μ* is the control parameter, and *u* and *v* are the changes of the image gray in the *x*- and *y*-directions, respectively. *f*(*x*, *y*)=−*E*_ext_′ is the edge mapping and ∇*f*=(*f*_*x*_, *f*_*y*_) is the edge gradient mapping.

Since the external force field of GVF is obtained through the principle of thermal diffusion, which is equivalent to multiscale Gaussian convolution, the Euler equation is calculated to solve the functional extremum in equation (7).

(8) $$\begin{array}{c} \left\{\begin{array}{c} \mu \nabla^{2}u-\left(u-f_{x}\right)\left(f_{x}^{2}+f_{y}^{2}\right)=0,\\ \mu \nabla^{2}v-\left(v-f_{y}\right)\left(f_{x}^{2}+f_{y}^{2}\right)=0. \end{array}\right. \end{array}$$

According to equation (8), the external force field of GVF can be obtained through multiple diffusions of ∇*f*. Therefore, the GVF snake model can solve the initialization problem of the traditional snake model and can initialize the contour to the inside or outside of the region of interest (ROI) while entering the “recessed” area of the image.

## 3. Research Methods

### 3.1. Data Acquisition

The experimental data in this study are all derived from the cardiac ultrasound images obtained by the transesophageal rotating ultrasound technology in the Department of Cardiology of Affiliated Hospital of Guangdong Medical University. The three-dimensional volume data of the cardiac ultrasound image is obtained after rotation. The cylindrical coordinates represent the three-dimensional volume data of cardiac ultrasound images. The interpolation method [16] is utilized to transform it into the form of the direct coordinate system, as illustrated in Figure 1. The interpolated three-dimensional volume data of the cardiac ultrasound image has a total of 23 data fields, each of which contains 231 tomographic images, and the size of the different tomographic images is 288 × 288. The cavity of the left ventricle is located between the 119th and 204th layers, so the size of the data field is set to 288 × 288 × 85 (*X* × *Y* × *Z*) in this study.

### 3.2. Construction of a Three-Dimensional Network Model of the Heart

In this study, the deformation model is employed to perform the three-dimensional segmentation processing of cardiac ultrasound images. Before the deformation processing, the initial contour of the heart needs to be obtained. Existing studies used the quadric surface to perform the fitting of the cardiac cavity model, which is then used for segmentation guidance [17]. However, the calculation of heart segmentation based on prior knowledge is very complicated. It is relatively simple to use the ellipsoid model to match the initial contour of the cardiac cavity, and the segmentation results also meet the requirements. Therefore, the ellipsoid model is employed to match the initial contour of the cardiac cavity. The main steps are as follows. First, the initial region growth method is adopted to perform ellipse matching of the middle-layer image of the test data field, and the initial matching result is shown in Figure 2(a). Second, with the center of the matching ellipse as the center of the ellipsoid, the *x*-axis, *y*-axis, and volume data layers of the ellipsoid are used as the *x*-axis, *y*-axis, and *z*-axis of the ellipsoid to match the ellipsoid, respectively, and the initial three-dimensional contour of the ellipsoid obtained by the matching is shown in Figure 2(b).

Deformation models have been widely used in the field of image segmentation. Compared with traditional image segmentation methods, the deformation model has segmentation results such as edge detection, target extraction, and 3D reconstruction. Moreover, the interactive operation method in the segmentation process can provide corresponding reference materials for the clinical diagnosis and pathological research of the disease [18–20]. The three-dimensional mesh model is the discretized expression form of the three-dimensional deformation model. It is improved based on the triangular mesh model and applied to the three-dimensional segmentation of cardiac ultrasound images. The discretization process of the ellipsoid model includes (i) sampling of the *xy*-plane of the ellipsoid, and the number of sampling points for each layer is set to 9, 18, 36, and 72 for processing. The results show that the number of sampling points is 36 when the effect is the best. Therefore, the number of sampling points for each layer is defined as 36 for subsequent experiments. (ii) Sampling points are connected on different layers in sequence. (iii) The sampling points at the same angle in adjacent layers are connected, and the discretized ellipsoid model is finally obtained.

### 3.3. Construction of a Three-Dimensional Deformation Model of the Heart

The three-dimensional deformation is processed based on the triangular mesh model of the initial contour of the ellipsoid constructed previously, which allows it to obtain an accurate cardiac cavity boundary under the combined action of internal and external forces, thereby realizing the three-dimensional segmentation of cardiac ultrasound images.

#### 3.3.1. Internal Force Calculation

The internal force *f*_in_ is the force that the model changes to the minimum position of the surface curvature *C*, which can maintain the smoothness and continuity of the active surface. The greater the curvature of the vertex, the greater the internal force moving to the smooth position. Therefore, the vertex curvature is solved first based on the basic element parameters of the triangle (Figure 3), and then the internal force of the deformation model is calculated. In Figure 3, *i* is the vertex, *D* is the connection vector from the vertex to the adjacent point, *d* is the unit connection vector from the vertex to the adjacent point, *n* is the unit normal vector of the triangle, and *r* is the normal vector of the vertex.

The specific steps for calculating the internal force are as follows:

(a) The first is the calculation of the unit normal vector of each triangle including the vertices. From Figure 3, the connection vector *D*_*i*,*j*_ between the vertex *i* and the adjacent point *A*(*i*, *j*) is defined as *D*_*i*,*j*_ = *x*_*i*_ − *x*_*A*(*i*,*j*)_, where *x* is the location of the vertex in the model position. The normalization processing of *D*_*i*,*j*_ can further obtain the unit connection vector *d*_*i*,*j*_ from vertex *i* to the adjacent point *A*(*i*, *j*), *d*_*i*,*j*_=*D*_*i*,*j*_/‖*D*_*i*,*j*_‖. The normal vector *N*_*i*,*j*_ of the triangular surface formed by vertex *i*, adjacent points *A*(*i*, *j*) and *A*(*i*, *j* + 1) is *N*_*i*,*j*_ = *d*_*i*,*j*_ × *d*_*i*,*j*+1_. Then, the unit normal vector *n*_*i*,*j*_=*N*_*i*,*j*_/‖*N*_*i*,*j*_‖. The triangle angle *θ*_*i*,*j*_ formed by vertex *i*, adjacent points *A*(*i*,*j*) and *A*(*i*, *j* + 1) is *θ*_*i*,*j*_ = cos^−1^(*d*_*i*,*j*_ × *d*_*i*,*j*+1_). The unit normal vector *r*_*i*,_ downward from vertex *i* is *r*_*i*_=*R*_*i*_/‖*R*_*i*_‖.
(b) The differences between the unit normal vector *r*_*i*,_ and the unit normal vector *n*_*i*,*j*_ of each triangle are calculated, and the weighted sum is used to determine the curvature *C*_*i*_ of the vertex *i*, which is calculated as follows:
  (9) $$\begin{array}{c} C_{i}=\frac{1}{\theta_{i,j}}\sum_{j=0}^{M_{i}-1}\theta_{i,j}\left\|r_{i}-n_{i,j}\right\|. \end{array}$$
(c) The unit normal vector *r*_*i*,_ of vertex *i* can determine the direction of internal force, and the curvature *C*_*i*_ of vertex *i* can determine the magnitude of internal force, so internal force *f*_in_ is defined as follows:
  (10) $$\begin{array}{c} f_{\mathrm{in},i}=\left|C_{i}-\frac{1}{M_{i}}\sum_{j=0}^{M_{i}-1}C_{A\left(i,j\right)}\right|r_{i}. \end{array}$$

#### 3.3.2. External Force Calculation

The GVF snake model can expand the distribution range of the external force field and improves the edge extraction of the “recessed” area to a certain extent. However, its edge extraction of “deep recessed area” still has defects [21], which may be due to the loss of some detailed information in the image while the GVF snake model expands the range of the external force field. Therefore, an improved method capable of extracting deep recessed areas vortical gradient vector flow (VGVF) snake model is proposed based on GVF snake model. The VGVF field is a composite field based on the GVF field combined with a constant vector as a cross product. Its biggest feature is that the direction of the force field rotates around the edge of the target.

The energy equation of the snake model is shown in equation (11). Assuming that *y*(*s*) is the effective solution of equation (11), which is defined as a movable *εσx*(*s*) range, then a new active contour curve is obtained.

(11) $$\begin{array}{c} y\left(s\right)+\varepsilon \sigma x\left(s\right)=\left\{y\left(s\right)+\varepsilon \sigma_{x}\left(s\right),\bar{\bar{u}}\left(s\right)+\varepsilon \sigma_{u}\left(s\right)\right\}. \end{array}$$

The general equation of the energy function is as follows:

(12) $$\begin{array}{c} E\left(y\left(s\right)+\varepsilon \sigma x\left(s\right)\right)=\int_{2}^{1}E_{\mathrm{int}}\left(y\left(s\right)+\varepsilon \sigma_{x}\left(s\right)\right)+E_{\mathrm{ext}}\left(y\left(s\right)+\varepsilon \sigma_{x}\left(s\right)\right)ds. \end{array}$$

In equation (11) and equation (12), *ε* is a nonzero infinitesimal scaling function.

Taylor's formula is used to expand the external energy function *E*_ext_ in equation (12), and then the following equation is obtained:

(13) $$\begin{array}{c} E_{\mathrm{ext}}\left(y\left(s\right)+\varepsilon \sigma_{x}\left(s\right)\right)=E_{\mathrm{ext}}\left(y\left(s\right),\bar{\bar{u}}\left(s\right)\right)+\varepsilon \sigma_{x}\left(s\right)\frac{\partial E_{\mathrm{ext}}}{\partial x}+\varepsilon \sigma_{y}\left(s\right)\frac{\partial E_{\mathrm{ext}}}{\partial y}. \end{array}$$

After derivation of equation (13), it is transformed into Euler's equation, and the following equation is obtained:

(14) $$\begin{array}{c} \alpha x^{\prime \prime }\left(s\right)-\beta x^{\prime \prime \prime }\left(s\right)-\nabla E_{\mathrm{ext}}=0. \end{array}$$

Formula (14) is the force balance equation; that is, *F*_int_ + *F*_ext_ = 0. Therefore, the internal force *F*_int_=*αx*^″^(*s*) − *βx*^‴^(*s*), and the external force *F*_ext_=−∇*E*_ext_. VGVF is used to perform work on the depression after the action of external force, and the maximum value of *W*=*F*_ext_ · *S* is finally obtained.

### 3.4. Solution of the Minimum Value of Energy Function

To reduce the computational complexity, the greedy algorithm [22] is employed to solve the minimum energy function. The mathematical expression of the energy function using the greedy algorithm is as follows:

(15) $$\begin{array}{c} E=\int \left(\alpha \left(s\right)E_{a}+\beta \left(s\right)E_{b}+\lambda \left(s\right)E_{c}\right)ds. \end{array}$$

In equation (15), *E*_*a*_ is the elastic potential energy of the profile curve, *E*_*b*_ is the curvature potential energy of the profile curve, *E*_*c*_ is the image potential energy of the profile curve, and *α*, *β*, and *λ* are parameters of equilibrium energy.

The mathematical expression of elastic potential energy in equation (15) is as follows:

(16) $$\begin{array}{c} E_{a}=\bar{d}-\left|v_{i}-v_{i-1}\right|=\bar{d}-\sqrt{{\left(x_{i}-x_{i-1}\right)}^{2}+{\left(y_{i}-y_{i-1}\right)}^{2}}. \end{array}$$

In equation (16), $\bar{d}$ is the average distance between adjacent control points on the boundary of the target contour, and |*v*_*i*_ − *v*_*i*−1_| is the distance between the control point and the critical point. When the greedy algorithm is used for calculation, the energy function reaches the optimum when $E_{a}=\bar{d}-\left|v_{i}-v_{i-1}\right|=0$, and at this time, the control points reach the average value.

The mathematical expressions of curvature potential energy and image potential energy in equation (15) are as follows:

(17) $$\begin{array}{c} E_{b}={\left|v_{i-1}-2v_{i}+v_{i+1}\right|}^{2}={\left(x_{i-1}-2x_{i}+x_{i+1}\right)}^{2}+{\left(y_{i-1}-2y_{i}+y_{i+1}\right)}^{2},\\ E_{c}={\left|\nabla \left[G_{\sigma }\left(x,y\right)*I\left(x,y\right)\right]\right|}^{2}. \end{array}$$

When most of the vertices on the active contour curve do not move, this indicates that the vertices on the curve have almost reached the minimum energy. Therefore, it is considered that the evolutionary convergence of the curve has reached the target boundary position.

### 3.5. Segmentation Processing of Cardiac Ultrasound Images

The proposed method is used to segment the cardiac ultrasound image. The segmentation process is shown in Figure 4. The main segmentation steps include the following: (i) three-dimensional volumetric data of cardiac ultrasound is acquired, and the initial model of the ellipsoid is matched to obtain the initial contour of the ellipsoid; (ii) the initial contour of the ellipsoid is discretized based on the triangular basic unit structure to obtain a triangular mesh model of the ellipsoid; (iii) the VGVF external force field is introduced, and deformation processing is done after the internal force and external force are calculated, so as to obtain the segmentation result; (iv) the final output segmentation result is the cardiac cavity structure.

Visual C++ programming software and OpenGL three-dimensional graphics software package are employed to build a three-dimensional segmentation platform for cardiac ultrasound images. Then, the three-dimensional display of the results of the cardiac cavity segmentation is performed, which facilitates the detection of changes in the cardiac cavity.

### 3.6. Evaluation Indexes of Segmentation Performance

To evaluate the performance of the VGVF snake model for ultrasonic image segmentation processing, area overlap rate (AOR) and mean contour distance (MCD) are measured.

AOR reflects the degree of overlap between the target contour extracted by the segmentation algorithm and the area contained in the real contour. The higher the AOR, the more similar the contour extracted by the segmentation algorithm is to the real contour. The calculation of AOR is as follows:

(18) $$\begin{array}{c} \mathrm{AOR}\left(x,y\right)=\frac{\mathrm{Area}\left\{C_{1}\cap C_{2}\right\}}{\mathrm{Area}\left\{C_{1}\cup C_{2}\right\}}\times 100\%. \end{array}$$

In equation (18), *x* and *y* are the contour extracted by the algorithm and the real contour, respectively, and *C*_1_ and *C*_2_ are the regions included in *x* and *y*, respectively.

MCD reflects the overall degree of overlap between the target contour extracted by the segmentation algorithm and the real contour (i.e., the difference in details of the contour). The larger the MCD, the greater the difference between the detailed information of the contour extracted by the segmentation algorithm and the real contour. The calculation of MCD is as follows:

(19) $$\begin{array}{c} \mathrm{MCD}\left(x,y\right)=\frac{1}{2}\left(\frac{\sum_{i=1}^{N_{x}}\mathrm{Dis}\left(\rho_{x}\left(i\right),y\right)}{N_{x}}+\frac{\sum_{j=1}^{N_{y}}\mathrm{Dis}\left(\rho_{y}\left(j\right),x\right)}{N_{y}}\right). \end{array}$$

In equation (19), *ρ*_*x*_ and *ρ*_*y*_ are points on the contour *x* and *y*, respectively; *N*_*x*_ and *N*_*y*_ are the number of points on the contour *x* and *y*, respectively; and Dis is the vertical distance from the point to the contour.

## 4. Research Results

### 4.1. Comparison of Segmentation Results of Different Models

First, different segmentation algorithms, snake model, GVF snake model, and VGVF snake model, are compared in terms of the convergence of the recessed area. The weighting coefficients *α* and *β* in the model are set to be 0.05 and 0.00, respectively. The maximum number of iterations of the model is set to 15. Then, each model is applied to the segmentation processing of the “U-shaped” image. The comparison of the experimental results is shown in Figure 5. The initial position is given on the U-shaped graph (Figure 5(b)), and the traditional snake model is adopted to extract the target contour. From Figure 5(c), the active contour curve extracted by the snake model cannot continue to move into the deep recessed area in the image, and the final contour stops at the entrance of the deep recessed area. From Figure 5(d), the direction of the external force field of the snake model at the depressed boundary of the target area is opposite to each other. The GVF snake model is utilized to extract the target contour. From Figure 5(e), the GVF snake model can perform target extraction in recessed areas to a certain extent, but cannot effectively extract deep recessed areas. From Figure 5(f), the external force field distribution range of the GVF snake model is slightly wider than that of the snake model. The VGVF snake model is used to extract the target contour. From Figure 5(g), the VGVF snake model can extract all target regions, including deep recessed areas. From Figure 5(h), the external force field of the VGVF snake model has a wide distribution range, and the external force of the VGVF snake model in the deep depression area has an obvious downward trend. The results show that the traditional snake model cannot effectively segment the recessed area, and the GVF snake model cannot segment the deep recessed area [23, 24].

### 4.2. Contour Extraction Test Results of Cardiac Ultrasound Images

Firstly, the effect of different segmentation algorithms, snake model, GVF snake model, and VGVF snake model, and doctor's manual extraction method to extract the left ventricle in cardiac ultrasound images is qualitatively evaluated. The results are shown in Figure 6, where the yellow dashed line is the segmentation result. The parameter settings of the snake model, GVF snake model, and VGVF snake model are as follows. The Gaussian standard deviation is 3, the balance coefficient is 0.2, the time step is 1, and the number of iterations of the external force vector field is 100. Due to the influence of false edges in the image, the result of the snake model for ventricular segmentation is not very satisfactory, and the control of the direction line is relatively rough. The GVF snake model for segmentation of the central ventricle in ultrasound images cannot achieve complete segmentation of the ventricular region, and the effect of segmentation for complex regions is not ideal. The reason may be that the false edges caused by the uneven grayscale of the ultrasound image affect the distribution of the GVF vector field, making the segmentation contour and the actual area contour different [25]. The segmentation results of the VGVF snake model proposed are basically similar to the manual segmentation results of physicians and can achieve effective segmentation in deep recessed areas. It shows that the VGVF snake model has an excellent weak edge convergence effect and can make up for the segmentation shortcomings of the GVF snake model. The VGVF snake model can obtain excellent segmentation results for images with uneven background grayscale and complex noise in the segmentation processing of ultrasound images versus the traditional snake model and GVF snake model, which lays the foundation for the subsequent quantitative assessment of the cardiac cavity.

With the doctor's manual segmentation result as the standard, a total of five standard curves are obtained in the same image. Subsequently, the AOR and MCD are measured to quantitatively evaluate the segmentation results of different models, and the results are shown in Figure 7. The snake model, GVF snake model, and VGVF snake model perform ultrasonic image segmentation with mean AOR of 20.50%, 38.52%, and 96.74%, and mean MCD of 61.24, 41.31, and 5.48, respectively. AOR evaluates the similarity between the algorithm segmentation area and the standard area. The larger the AOR, the higher the overlap between the area and the standard area after algorithm segmentation. MCD evaluates the degree of coincidence between the contour curve of the algorithm segmentation and the contour curve of the standard area. The smaller the MCD is, the closer the contour curve of the algorithm segmentation is to the contour curve of the standard area. The results show that the AOR of VGVF snake model for ultrasonic image segmentation is dramatically superior to the traditional snake model and GVF snake model, which exceeds 95%. MCD of VGVF snake model for segmentation of ultrasound images is greatly lower than that of snake model and GVF snake model, which is only 5.48. The above results show that the VGVF snake model has high-efficiency performance in ultrasonic image segmentation processing.

### 4.3. Two-Dimensional Projection of Cardiac Ultrasound Images Based on Segmentation Results of Deformed Models

The differences of the results of the ultrasound image segmentation are compared between the proposed VGVF snake deformation model under ellipsoid contour and the manual segmentation of the doctor. The results are shown in Figures 8 and 9. The segmentation results of the proposed model for ultrasound images are basically similar to the manual segmentation standard results and generally meet the segmentation requirements. The ellipsoid contour VGVF snake deformation model used for the segmentation of cardiac ultrasound images can clearly express the size, shape, and position of the cardiac cavity, which also solves the problem of selecting the initial contour of the model. The attraction range of the object boundary to the active contour is increased, and the segmentation processing of the boundary of the deep recessed area is realized.

The cardiac cavity obtained by segmentation of the ellipsoid contour VGVF snake deformation model still have certain differences in detail at the edge of the recessed area in contrast to the standard result of manual segmentation. It may be because there is a lot of speckle noise in the ultrasound image, which causes the VGVF snake model to fall into the local minimum area caused by speckle noise, and it ultimately affects the segmentation effect of the model [9].

The difference between the ellipsoid contour VGVF snake deformation model for cardiac ultrasound image segmentation and the doctor's manual segmentation is quantitatively evaluated regarding the AOR and MCD, and the results are shown in Figure 10. The average AOR is 97.4%, and the average MCD is 3.2. It shows that the proposed ellipsoid contour VGVF snake deformation model used for the segmentation of the central ventricle of the cardiac ultrasound image has a close similarity with the ventricular region and the region contour manually segmented by the doctor, which meets the image segmentation requirements.

### 4.4. Quantitative Measurement of Cavity Volume Based on Cardiac Ultrasound Image Segmentation

OpenGL is employed to perform the three-dimensional display of the cardiac cavity image after segmentation of the ellipsoid contour VGVF snake deformation model, and the result is shown in Figure 11. The ellipsoid contour VGVF snake deformation model is adopted to segment the cardiac cavity in the cardiac ultrasound image. Then, a triangular mesh model of the cardiac cavity is built, as illustrated in Figure 11(a). The surface rendering of the cavity is performed based on the triangular mesh model of the cardiac cavity (Figure 11(b)).

A quantitative measurement of the volume of three different heart cavities in a cardiac cycle is performed based on the segmentation result of the cardiac cavity, and the measurement result is shown in Figure 12. In a cardiac cycle, the volumes of different left ventricles all show a trend of increasing to decreasing to increasing. The volumes of different left ventricles all reach the largest at the 3rd frame and reach the lowest at the 14th frame. The changing trend of different left ventricular volume is basically the same.

## 5. Conclusion

The ellipsoid model is utilized to segment the initial contour of the cardiac ultrasound image, so as to improve the segmentation effect of the cardiac ultrasound image and realize the quantitative measurement of the volume of the cardiac cavity. Based on which, the VGVF external force field and greedy algorithm are introduced to process the deformation of the initial contour of the cardiac ultrasound image. After comparison, it is found that the results of the proposed model for cardiac ultrasound image segmentation are closer to the manual segmentation results relative to those of the traditional snake and GVF snake models. In addition, the quantitative measurement of the cavity volume change is realized based on the segmentation result of the cardiac cavity. This study only explores the differences in segmentation effects among different segmentation algorithms, but does not consider the effects of artifacts and noise in ultrasound images on the segmentation results. Therefore, the follow-up work will further combine denoising, segmentation, feature extraction, and other methods to build an intelligent diagnosis and treatment system for cardiovascular diseases, to provide a basis for improving the diagnosis rate and treatment rate of cardiovascular diseases in clinical diagnosis.

## Figures and Tables

**Figure 1:** Three-dimensional volume data conversion of cardiac ultrasound images based on interpolation.

**Figure 2:** Ellipse fitting based on initial area growth (a) and three-dimensional initial contour fitting of ellipsoid (b).

**Figure 3:** Triangular basic unit parameters.

**Figure 4:** The segmentation process of the cardiac cavity. *Note*. The yellow fill is the introduced VGVF snake model.

**Figure 5:** U-shaped contour extraction results of different segmentation algorithms. (a) The original image; (b) initial contour marking based on ellipse model; (c) the contour extracted by the snake model; (d) the external force field distribution of the snake model; (e) the contour extracted by the GVF snake model; (f) the external force field distribution of the GVF snake model; (g) the contour extracted by the VGVF snake model; (h) the external force field distribution of the VGVF snake model.

**Figure 6:** Comparison of the effect of different models for segmentation of cardiac ultrasound images. (a) Original echocardiogram; (b) snake model segmentation results; (c) GVF snake model segmentation results; (d) VGVF snake model segmentation results; (e) doctor manual segmentation results; the yellow dashed line is the segmentation result.

**Figure 7:** Comparison of AOR and MCD of ultrasound images processed by different models.

**Figure 8:** Heart ultrasound segmentation results of the ellipsoid contour VGVF snake deformation model (the yellow dotted line in the figure is the segmentation result of the VGVF snake model).

**Figure 9:** Heart ultrasound segmentation results manually segmented by the doctor (the red dotted line in the figure is the result of manual segmentation by the doctor).

**Figure 10:** AOR and MCD of ellipsoid contour VGVF snake deformation model segmenting ultrasound images.

**Figure 11:** Three-dimensional display of the segmentation results of the cardiac cavity. (a) The triangular mesh model of the cardiac cavity. (b) The surface rendering result of the cardiac cavity.

**Figure 12:** The volume change of the left ventricle based on the segmentation result of the cardiac cavity. (a) Heat map of left ventricular volume change. (b) Left ventricular volume versus time curve.

## Data Availability

No data were used to support this study.
